# P38 Plays an Important Role in Glucolipotoxicity-Induced Apoptosis in INS-1 Cells

**DOI:** 10.1155/2014/834528

**Published:** 2014-03-05

**Authors:** Lingli Zhou, Xiaoling Cai, Xueyao Han, Linong Ji

**Affiliations:** Department of Endocrinology and Metabolism, Peking University People's Hospital, Beijing 100044, China

## Abstract

*Objectives*. The mechanism underlying the regulation of glucolipotoxicity-induced apoptosis by MAPKs was examined in INS-1 cells. *Methods*. The rat insulinoma cell line INS-1 was cotreated with glucose (30 mM) and palmitic acid (0.2 mM) (GLU+PA). Apoptosis was assessed by cell morphology and detection of PARP cleavage. The activation of MAPKs was examined by Western blotting using specific antibodies against the phosphorylated forms of JNK, ERK1/2, and P38. *Results*. (1) Live cell imaging studies showed that treatment with GLU+PA for 72 h induced significant cell death, concomitant with PARP-1 cleavage and caspase-3 activation, which peaked at 96 h of treatment. (2) Western blot analysis of the activation of MAPKs during GLU+PA-induced INS-1 cell apoptosis showed that phosphorylation of P38 increased gradually and reached a peak at 96 h, which coincided with PARP-1 cleavage. A transient increase of ERK activation was followed by a rapid decline at 96 h, whereas JNK phosphorylation status remained unchanged in response to GLU+PA. (3) Phosphorylation of insulin receptor substrate (IRS)-2 at 48 h of treatment triggered its degradation, which coincided with P38 activation. (4) Inhibition of P38, but not JNK or ERK, blocked GLU+PA-induced INS-1 cell apoptosis. *Conclusions*. P38 may be involved in the regulation of glucolipotoxicity-induced apoptosis through the phosphorylation of IRS-2.

## 1. Introduction

Type 2 diabetes (T2DM) is a complex disease characterized by chronic hyperglycemia. Beta cell dysfunction and insulin resistance are the main pathogenetic factors associated with T2DM [1]. The evolution of T2DM is characterized by a progressive decline of *β*-cell function that leads to the failure of oral antidiabetic therapy at controlling glucose levels and a requirement for insulin injections. However, insulin resistance generally existed for a long period before diagnosis of T2DM and remains unchanged after diagnosis, indicating that *β*-cell function might play a more important role in progressive hyperglycemia. Analyses of human pancreases obtained by autopsy showed decreased *β*-cell volume in individuals with T2DM compared to nondiabetic controls. The frequency of *β*-cell replication was very low in all cases, and neogenesis was similar in diabetic and nondiabetic groups. However, there was a striking increase in *β*-cell apoptosis in the diabetic subjects compared to their respective controls [2]. This suggests that in T2DM, acceleration of *β*-cell apoptosis is not compensated by a matched increase in *β*-cell replication. Although the pathogenesis of *β*-cell decompensation associated with insulin resistance has not been elucidated, endoplasmic reticulum stress and oxidative stress caused by increased levels of glucose or free fatty acids (FFA) contribute to the deterioration of *β*-cell function. The effects of glucose and FFA on *β*-cell dysfunction have been studied extensively in the last 20 years. Prolonged exposure to elevated levels of glucose or FFAs is associated with induction of apoptotic cell death, termed “glucotoxicity” or “lipotoxicity” [3, 4]. Several lines of evidence indicate that lipotoxicity only occurs in the presence of a concomitant increase in glucose levels. Thus, the term “glucolipotoxicity” is now widely accepted to describe the synergistic effects of elevated glucose and lipids on *β*-cell dysfunction [5–7]. However, the molecular mechanisms linking glucolipotoxicity to *β*-cell dysfunction remain poorly understood. Therefore, the investigation of this biologic pathway and the identification of drug targets for the design of therapies aimed at protecting *β*-cell function and suppressing the development of T2DM are critical.

Mitogen-activated protein kinases (MAPKs) play pivotal roles in cell survival, apoptosis, proliferation, and differentiation. MAPKs subfamilies include three members, ERKs, JNK, and P38. ERKs mainly regulate cell survival and proliferation, whereas JNK and P38 have been associated with cell death and stress responses [8]. Elevated glucose or FFA activates MAPK signaling cascades; however, the function of MAPKs in glucotoxicity and lipotoxicity remains controversial. Some studies suggest that JNK activation is associated with high levels of glucose-induced apoptosis. However, under certain conditions, JNK is a survival signal in response to stress [9, 10]. In the present study, the rat INS-1 *β*-cell line was treated with high levels of glucose (GLU) and palmitic acid (PA) to induce apoptotic cell death, and the role of MAPKs in regulating GLU+PA-induced apoptosis of *β*-cells was investigated. We showed, for the first time, that GLU+PA-induced apoptosis occurs through a mitochondrial-dependent pathway, and that P38 plays an important role in the regulation of GLU+PA-induced apoptosis in INS-1 cells.

## 2. Materials and Methods

### 2.1. Chemicals and Reagents

Rabbit anti-phospho-JNK, rabbit anti-phospho-ERK, and rabbit anti-phospho-P38 monoclonal antibodies; rabbit anti-insulin receptor substrate (IRS)-2 and goat anti-PARP-1 polyclonal antibodies; and rabbit anti-*β*-actin antibody were purchased from Santa Cruz Biotechnology, CA, USA. PD98059 was from Cell Signaling, Beverly, MA, USA, and palmitate was obtained from Sigma, Louis, MO, USA. SB203580 and SP600125 were from Calbiochem, San Diego, CA, USA. Hoechst33342 was from Molecular Probes. Glucose (50%) was from Tianjing pharmaceutical of Group (Jiaozuo) Ltd., Tianjing province, China.

### 2.2. Preparation of PA Solution

Palmitate powder (0.1025 g) was dissolved in 1 mL of 400 mM NaOH for 30 min at 70°C. The solution was shaken until clear and then sterilized by filtration. A volume of 1 mL of the solution was added to 7 mL of 10% fatty acid-free bovine serum albumin and shaken at 55°C. The stock solutions were finally titrated to 50 mM at PH 7.2–7.4 and stored at −80°C.

### 2.3. Cell Culture and Induction of Apoptosis

Rat INS-1 cell lines were a kind gift from Professor Yang Wenying (China-Japan Friendship Hospital). INS-1 cells were grown in RPMI 1640 medium with 11.2 mM glucose supplemented with 10% fetal bovine serum, 10 mM HEPES, 2 mM L-glutamine, 1 mM sodium pyravate, 50 µM *β*-mercaptoethanol, 100 U/mL penicillin, and 100 mg/mL streptomycin at 37°C. INS-1 cells used in the present study were harvested at passages 16−23. Cell images were obtained using a phase-contrast microscope (IMT-2, Olympus, Tokyo, Japan) equipped with a digital camera. Cells were plated on glass coverslips and 24 h later, cells were exposed to glucose (30 mM) and PA (0.2 mM).

### 2.4. Fluorescent Immunostaining

INS-1 cells grown on coverslips were treated with GLU+PA. Cells were fixed at different time points with 4% paraformaldehyde plus 0.1% glutaradehyde for 15 min at room temperature, and then rinsed 3 times in PBS, permeabilized with 0.2% Triton X-100 in PBS for 15 min, and then blocked in 3% BSA in PBS at 4°C for overnight. After blocking, cells were incubated with mouse anti-native Cytochrome c (1 : 200 dilution in 3% BSA) antibody at 4°C for overnight. Then cells were stained with secondary antibody which is goat anti-mouse conjugated with FITC (1 : 200 dilution).

### 2.5. Real-Time Polymerase Chain Reaction

Total RNA of cells was extracted with TRIZOL reagents (Invitrogen, Carlsbad, CA). Real-time PCR was carried out with SYBR green PCR Master Mix (TOYOBO) as described by the manufacturer to measure IRS-2 mRNA (forward, 5′-CTACCCACTGAGCCCAAGAG-3′ and reverse, 5′-CCAGGGATGAAGCAGGAC-3′) relative to *β*-actin mRNA (forward, 5′-GACAGGATGCAGAAGGAGATTACT-3′ and reverse, 5′-TGATCCACATCTGCTGGAAGGT-3′). All samples were run in duplicate on a 7300 Sequence Detection System (Applied Biosystems, Foster City, CA).

### 2.6. Western Blot Analysis

INS-1 cells were cultured in 100 mm Petri dishes. Cells were harvested at different time points after treatment with 30 mM glucose and 0.2 mM palmitate and lysed in NP-40 lysis buffer (50 mM Tris-HCL, PH 8.0, 150 mM NaCL, and 1% NP-40) in the presence of protease inhibitors. Whole cell lysates (100 µg/lane) were separated on 10% SDS-PAGE followed by electrophoretic transfer onto nitrocellulose membranes (Amersham Pharmacia, Piscataway, NJ). Membranes were probed (or reprobed) with specific antibodies at a dilution of 1 : 1000 for 3 h at room temperature. The membranes were incubated with horseradish peroxidase-conjugated secondary antibody at a dilution of 1 : 5000 for 1 h and developed using the ECL Western blotting analysis system.

### 2.7. Cell Imaging

The fixed cells were examined by a fluorescence microscope using a 40 × oil or 100 × oil objective. Laser line of 488 nm and 365 nm was used to observe FITC conjugated antibody and Hoechst stained cell nuclei, respectively. Cells with condensed but fragmented chromosomes were considered as apoptotic cells. To count apoptotic cells, at least 10 fields and more than 100 cells for each time point were examined. We used the MetaMorph v6.0 software (Universal Image, West Chester, PA) to analyze digital images. Quantity One Software was used to quantify the targeted bands on western-blot.

### 2.8. Statistical Analysis

All values are presented as Means ± SD. Comparisons among groups were analyzed by ANOVA. *P* < 0.05 was considered statistically significant.

## 3. Results

### 3.1. Combination Treatment with High Concentrations of Glucose and PA Induces Apoptosis in INS-1 Cells

To examine the effect of combination treatment with high concentrations of glucose and PA on pancreatic *β*-cells, rat pancreatic INS-1 cells were exposed to 30 mM glucose and 0.2 mM PA. Live cell imaging showed that GLU+PA had a negative effect on INS-1 cell adherence. As shown in Figure 1(a), most GLU+PA treated cells were detached from the Petri dish and floated in the medium at 96 h after treatment.

To determine whether GLU+PA treatment induces apoptotic cell death in INS-1 cells, PARP-1 cleavage was assessed by Western blotting in cells treated with GLU+PA and harvested at different time points. The cleaved fragment of PARP-1 (approximately 25 kDa) was detected at 72 h after GLU+PA treatment and its level increased with time, whereas the full-length PARP-1 (approximately 113 kDa) decreased with time (Figure 1(b)). In addition, caspase-3 activity increased with time (Figure 1(c)) and cytochrome c, which is released from mitochondria during the early stages of apoptosis, was detected in the cytosol after treatment (Figure 1(d)). These data suggest that GLU+PA induces mitochondrial-dependent apoptosis in INS-1 cells.

INS-1 cells were grown on 100 mm Petri dishes and cotreated with 30 mM glucose and 0.2 mM palmitate. (a) Cell morphology was assessed by phase-contrast microscopy. Images were obtained at different treatment time points with a digital camera. (b) Cells were harvested at 0, 24, 48, 72, and 96 h of GLU+PA treatment. Cell lysates were analyzed by 10% SDS-PAGE and immunoblotting against anti-PARP-1 antibodies. Beta-actin was used as a loading control. (c) INS-1 cells were treated with GLU+PA for the indicated times. Cell extracts were prepared and used for caspase-3 activity assay as described in Materials and Methods. (d)INS-1 cells were treated with 0.5% DMSO (control) or GLU+PA for 72 h, immunostained with an anticytochrome c antibody, and visualized by indirect immunofluorescence.

### 3.2. P38 Is Activated during Glucolipotoxicity-Induced Apoptosis

To explore the involvement of MAPKs in *β*-cell apoptosis, the phosphorylated forms of JNK, ERK1/2, and P38 were detected by Western blotting with specific antibodies to determine the activation status of these MAPKs in response to treatment. As shown in Figure 2, GLU+PA treatment resulted in the transient activation of ERK between 24 and 48 h after treatment. The levels of phospho-ERK started to decline at 72 h and became undetectable at 96 h. However, the level of activated JNK remained unchanged during the course of GLU+PA treatment. The level of phosphorylated P38, which was low in untreated INS-1 cells, gradually increased at 24 h and reached a peak value at 96 h after GLU+PA treatment.

To determine whether MAPKs play a role in GLU+PA-induced apoptosis, cells were treated with specific inhibitors of JNK, P38, and MEK. As shown in Figure 3, the P38 inhibitor SB203580 reversed the cytotoxic effect of GLU+PA on INS-1 cells. However, the MEK inhibitor PD98059 and the JNK inhibitor SP600125 had no effect on GLU+PA-induced cell death.

### 3.3. Phosphorylation and Degradation of Insulin Receptor Substrate-2 during Glucolipotoxicity-Induced Apoptosis

P38 has been proposed to exert its proapoptotic effects through the phosphorylation of apoptotic regulators such as Bcl-2 family proteins. Here, we examined the phosphorylation status of the antiapoptotic protein IRS-2 during GLU+PA-induced apoptosis. As shown in Figure 4, mRNA levels of IRS-2 increased during GLU+PA treatment; however, the protein levels of IRS-2 decreased dramatically at 96 hr after treatment. Furthermore, the phosphorylation of IRS-2 was detected at 48 h and became obvious at 72 h after GLU+PA treatment, as indicated by the slow migrating bands on SDS-PAGE. The levels of phosphorylated IRS-2 became undetectable at 96 h of treatment, indicating the degradation of the antiapoptotic protein IRS-2 during GLU+PA-induced apoptosis. Comparison of the time course of IRS-2 phosphorylation and P38 activation suggested that IRS-2 phosphorylation is temporally correlated with P38 activation.

## 4. Discussion

The induction of pancreatic *β*-cell dysfunction by high levels of lipids or glucose has been well documented in numerous *in vitro* experimental systems. Several studies have provided evidence that elevated glucose concentration alone is not toxic to islet tissue in normal or prediabetic stages, and lipotoxicity only occurs in the presence of concomitantly elevated glucose levels. Furthermore, patients with type 2 diabetes often show high glucose and lipid levels simultaneously. High glucose level (11–30 mM) has traditionally been used to generate the glucotoxicity model, whereas high palmitate (0.2 mM) is used in the lipotoxicity model. However, an experimental model of glucolipotoxicity remains to be established. In the present study, we treated INS-1 cells with 30 mM glucose and 0.2 mM palmitate to induce glucolipotoxicity. Combination treatment with glucose and PA at these concentrations induced apoptosis of INS-1 cells. Furthermore, our results showing the release of cytochrome c from mitochondria into the cytosol and caspase-3 activation indicated that the combination GLU+PA induced mitochondrial-dependent apoptotic cell death in INS-1 cells.

MAPK-dependent signaling pathways are known to be involved in *β*-cell dysfunction. In the present study, MEK/ERK1/2 was early and transiently activated during GLU+PA-induced apoptosis. Consistent with previous studies showing the role of MEK/ERK1/2 as survival signals, treatment of cells with MEK inhibitors promoted GLU+PA-induced apoptosis in INS-1 cells in the present study. However, the roles of JNK and P38 during apoptosis have remained controversial. Several studies have indicated that JNK and P38 promote *β*-cell apoptosis, whereas other studies suggest that JNK and P38 may exert a prosurvival effect. This discrepancy could be attributed to the use of different cell types and stimuli. In previous studies, high concentrations of glucose or FFA were used to induce *β*-cell apoptosis. However, neither glucose nor FFA alone is capable of causing clinically significant *β*-cell toxicity, especially in patients with normal or impaired glucose tolerance. Because high glucose acts synergistically with FFAs to stimulate *β*-cell apoptosis, combination treatment with high concentrations of glucose and FFA is a more accurate method to mimic the physiological diabetic condition. In this experimental system, exposure to a JNK inhibitor did not affect GLU+PA-induced apoptosis. However, the activation of P38 during apoptosis induction and the suppression of apoptosis by a P38 inhibitor suggested that P38 is indeed involved in GLU+PA-induced apoptosis. To our knowledge, this is the first study to show the role of P38 during GLU+PA-induced apoptosis.

P38 has long been postulated as an attractive therapeutic target for atherosclerosis because of its critical role in the generation and transduction of proinflammatory cytokine signaling [11]. Recent studies have suggested an association between type 2 diabetes and inflammation [12]. Inflammation is present prior to the development of T2D and cardiovascular disease (CVD), supporting the “common soil” hypothesis, which is a reference to the common risk factors for the development of these two diseases [13]. The Multi-Ethnic Study of Atherosclerosis showed that higher levels of the inflammatory markers, C-reactive protein and interleukin-6, were associated with an increased risk of developing T2D [14]. These proinflammatory molecules activate the cells of innate immunity, resulting in damage to tissues in the vasculature, adipose tissue, and pancreas. Hyperglycemia and hyperlipidemia are significant stressors that have also been shown to cause chronic inflammation and contribute to the pathogenesis of T2D [15]. P38, which contributes to the pathogenesis of diabetic nephropathy, is activated in *in vivo* glomeruli from diabetic rats and in mesangial cells exposed to high glucose. Early intensive insulin treatment prevents the increase in renal cortical P38 activity in diabetic rats, thereby attenuating the pathological changes associated with diabetic nephropathy [16]. These results suggest that P38 could be a therapeutic target for diabetes.

The mechanisms underlying the deleterious effects of P38 on *β*-cells remain unclear. In the present study, we observed similarities in the temporal pattern of P38 activation and IRS-2 phosphorylation, leading to the assumption that P38 may contribute to IRS-2 phosphorylation. Our results suggested that inhibition of P38 activity attenuates INS-1 cell death by preventing the phosphorylation and degradation of IRS-2. Further studies are necessary to verify the direct phosphorylation of IRS-2 by P38.

Taken together, our results indicate that GLU+PA-induced apoptosis is mediated by the activation of P38 and the consequent phosphorylation of a variety of substrates, possibly including IRS-2. Phosphorylated IRS-2 is degraded, resulting in the reduction of its antiapoptotic effect. Inhibition of P38 prevents glucolipotoxicity in pancreatic *β*-cells* in vitro*. Our findings provide evidence supporting the use of P38 inhibitors as potential new therapeutic agents for the preservation of *β*-cell mass and function.

## Figures and Tables

**Figure 1:** GLU+PA treatment induces mitochondrial-dependent apoptosis in INS-1 cells.

**Figure 2:** Time course of MAPK activation in response to GLU+PA treatment in INS-1 cells. INS-1 cells were cotreated with 30 mM glucose and 0.2 mM palmitate and MAPK activation status was analyzed by Western blotting with anti-phospho-JNK, -P38, or -ERK antibodies.

**Figure 3:** Effect of preincubation with MAPK inhibitors on GLU+PA-induced apoptosis of INS-1 cells. (a) INS-1 cells were grown on 60 mm coverslips and preincubated with MAPK inhibitors (JNK: SP60015, P38: SB 203580, ERK: PD98059) before GLU+PA treatment. Cell morphology was examined and images were acquired by phase-contrast microscopy. (b) The cells were fixed and stained with Hoechst 33342 and at 96 h after GLU+PA treatment. The apoptotic percentages were calculated. **Comparing to control (only DMSO was added into GLU+PA-treated cells), *P* < 0.01 (ANOVA).

**Figure 4:** Effect of GLU+PA treatment on IRS-2 expression. INS-1 cells were cotreated with 30 mM glucose and 0.2 mM palmitate. Cells were collected at 0-, 24-, 48-, 72-, and 96 h after treatment. (a) The relative mRNA levels of IRS-2 were measured. The value obtained in 0 hr was considered as 1. The data was based on three independent experiments. *Comparing to control (0 h), *P* < 0.05 (ANOVA). (b) The cell extracts were analyzed by 10% SDS-PAGE followed by immunoblotting with antibodies against IRS-2. *β*-actin was used as a loading control. (c) The bars represented densitometric values normalized by *β*-actin. The value obtained in 0 hr was considered as 1. *Comparing to control (0 h), *P* < 0.05 (ANOVA).
